# Efficacy and safety of acupuncture therapy for asymptomatic infection of COVID-19: A protocol for systematic review and meta-analysis

**DOI:** 10.1097/MD.0000000000022697

**Published:** 2020-10-09

**Authors:** Shaolei Huang, Suyao Wang, Guoqiang Li, Mengmeng Wang, Wenjie Yu, Guoliang Shao, Jian Zhang, Dianhui Yang

**Affiliations:** a Shandong University of Traditional Chinese Medicine; b People's Hospital of Lixia District; c The First Affiliated Hospital of Shandong First Medical University, Jinan; d Weifang Hospital of Traditional Chinese Medicine, Weifang; e Affiliated Hospital of Shandong University of Traditional Chinese Medicine, Jinan, Shandong, China.

**Keywords:** acupuncture, asymptomatic infection of COVID-19, protocol, systematic

## Abstract

**Background:**

The study aims to evaluate the effectiveness and safety of acupuncture therapy for asymptomatic infection of COVID-19.

**Methods:**

The following electronic databases will be searched from December 2019 to December 2020: MEDLINE, PubMed, EMBASE, Web of Science, China National Knowledge Infrastructure (CNKI), Wan-fang database, Chinese Scientific Journal Database (VIP), Chinese Biomedical Literature Databases (CBM), and other databases. All published randomized controlled trials (RCTs) about this topic will be included. Two independent researchers will operate article retrieval, duplication removing, screening, quality evaluation, and data analyses by Review Manager (V.5.3.5). Meta-analyses, subgroup analysis, and/or descriptive analysis will be performed based on the included data conditions.

**Results:**

High-quality synthesis and/or descriptive analysis of current evidence will be provided from the time of negative nucleic acid detection for 2 consecutive times (not on the same day), cure rate, converting to clinical diagnosis rate, and side effects of acupuncture.

**Conclusion:**

This study will provide the evidence of whether acupuncture is an effective and safe intervention for asymptomatic infection of COVID-19.

**PROSPERO registration number:**

CRD 42020179729.

## 1 Introduction

### 1.1 Description of the condition

Since its emergence in December 2019, Coronavirus Disease 2019 (COVID-19) has spread rapidly around the world and become a serious public health event endangering human life.^[1–3]^ The main symptoms of COVID-19 are fever, dry cough, fatigue, and ground-glass opacities on computed tomography.^[4–6]^ As the epidemic is gradually brought under control, asymptomatic infections are also becoming a concern.^[7–10]^ COVID-19 asymptomatic infections refer to those who have no clinical symptoms but positive detection of novel coronavirus pathogens in respiratory specimens.^[11]^ They are mainly detected through screening of close contacts of confirmed patients. Asymptomatic infections may also become the contagious source of novel coronavirus, and have risk of transmission.^[12,13]^ There is no definitive treatment for them other than isolation and observation.^[14,15]^

### 1.2 Description and function of intervention

Acupuncture is an important part of traditional Chinese medicine and has been used as an important complementary therapy in the word. It treats diseases through the conduction of meridians and acupoints adding certain operations. Acupuncture therapies include many different treatments, such as acupuncture, moxibustion, electroacupuncture, fire needle, acupoint injection, auricular point therapy, etc. Acupuncture has been proved effective in some respiratory diseases.^[16–18]^ During the period of COVID-19, the China Association of Acupuncture-Moxibustion recommends acupuncture therapy for the treatment of COVID-19 including asymptomatic infections.^[19]^ Acupuncture therapy, especially moxibustion, is of great significance for the prevention of COVID-19 and treatment of asymptomatic infections.^[20,21]^

### 1.3 Why the review is important.

According to the published research, there is a lack of high-quality evidence on acupuncture in the treatment of COVID-19 asymptomatic infection. Therefore, this systematic review aims to assess the effectiveness and safety of acupuncture therapy for asymptomatic infection of COVID-19.

## 2 Methods

This systematic review protocol has been registered in the PROSPERO network (No. CRD42020179729). All steps of this systematic review will be performed according to the Cochrane Handbook (5.2.0).

## 3 Selection criteria

### 3.1 Types of studies

Randomized controlled trials (RCTs) of acupuncture therapy for asymptomatic infection of COVID-19 without any limitation of blinding or publication language will be included. RCTs that involve at least 1 acupuncture-related treatment to asymptomatic infection of COVID-19, and 1 control treatment (or blank treatment) will be included. The studies of animal experiment, review, case report, meta-analysis, and duplicate publications will be excluded.

### 3.2 Types of patients

Patients who were diagnosed as asymptomatic infection of COVID-19 will be included, without limits on gender, age, race, and nationality.

### 3.3 Types of interventions and comparisons

Interventions can be any type of acupuncture therapy: acupuncture, moxibustion, electroacupuncture, fire needle, acupoint injection, auricular point therapy. Multiple control interventions will be included: no treatment, placebo, and other interventions (e.g., standard care, drugs, Chinese medicine). Comparisons contain acupuncture and its relation will be excluded. Interventions of acupuncture combined with other therapies will also be included, only if the other therapies were used as comparisons.

### 3.4 Types of outcomes

Primary outcomes will include the time of negative nucleic acid detection for 2 consecutive times (not on the same day) and cure rate. Secondary outcomes will include converting to clinical diagnosis rate and side effects of acupuncture.

### 3.5 Search methods for identification of studies

#### 3.5.1 Electronic searches

The following electronic databases will be searched from December 2019 to December 2020: MEDLINE, PubMed, EMBASE, Web of Science, China National Knowledge Infrastructure (CNKI), Wan-fang database, Chinese Scientific Journal Database (VIP), Chinese Biomedical Literature Databases (CBM), and other databases. All published RCTs about this topic will be included. Exemplary search strategy of MEDLINE is listed in Table 1. According to the difference of databases, keywords may combine with free words and comprehensive search will be performed.

**Table 1:** MEDLINE search strategy.

### 3.6 Data collection and analysis

#### 3.6.1 Selection of studies

Two reviewers (SLH and SYW) will independently select the studies. They will check the results with each other. When disagreements occur, a third reviewer (GLS) will make the final decision. They will read the full texts of all included studies if necessary. Screening operation will flow the diagram of Figure 1. If the full literatures are unable to be obtained or related data are incomplete, we will contact the corresponding author.

**Figure 1:** Flow diagram of studies identified.

#### 3.6.2 Assessment and quality of included studies

Two reviewers (MMW and GQL) will evaluate quality of included articles and assess the risk of bias based on Cochrane Handbook 5.2.0. Quality assessment of included studies contains randomized method, allocation concealment, blinding of participants and personnel, blinding of outcome assessment, completeness of outcome data, and selective reporting. Divergence of evaluation will also consult a third reviewer (GLS).

#### 3.6.3 Data extraction

Two independent reviewers (SLH and WJY) will extract data after selection and quality assessment; they will extract the data using a standardized data extraction form and any differences of opinion between them will be resolved through discussion; if failed, they will discuss with the third reviewer (GLS). Data will be recorded onto an electronic form, including the basic information of the article (the title of article, first author, year, and language), inclusion and exclusion criteria, the baseline of the study (the sample size, sex ratio, and age), interventions in the observation group and the control group, and outcome measures.

#### 3.6.4 Measures of treatment effect

Two reviewers (SLH and SYW) will perform analysis independently and then cross-check treatment effect with Review Manager 5.3.5. Risk ratio (RR) with 95% confidence intervals (CIs) will be adopted when dichotomous data existence. Continuous data will be presented by mean difference (MD) or standard mean difference (SMD) with 95% CI. RR form will be changed to analyze when binary data existence.

#### 3.6.5 Dealing with missing data

Due to the possibility of data loss in the literature, we will contact the corresponding author by email or other means. If the missing data are not available, we will analyze the existing data assumed to be lost at random.

#### 3.6.6 Assessment of heterogeneity

The heterogeneity of studies will be evaluated by Q-test and *I*^2^ statistic with RevMan5.3.5. The heterogeneity will be deemed as low (*I*^*2*^ < 50%), moderate (50–75%), and high (*I*^*2*^ > 75%).

#### 3.6.7 Assessment of reporting bias

Publication bias and other reporting bias will be assessed by creating funnel plots. A symmetrical funnel plot indicates a low risk of bias, while an asymmetric funnel plot indicates a high risk of bias.

#### 3.6.8 Data synthesis

Meta-analysis or descriptive analysis will be conducted according to the intervention method, measurement method, and heterogeneity level. If clinical and methodological heterogeneity are low, the fixed-effect model with merger analysis will be used. When heterogeneity is at medium level, the random-effects model with merger analysis will be used. However, if the heterogeneity is significantly high, subgroup analysis or descriptive analysis will be performed.

#### 3.6.9 Subgroup analysis

Subgroup analysis will be performed based on the results of data synthesis, and if heterogeneity is found to be caused by the specific characteristics of the included study (e.g., age, the intervention methods, and the measurement methods used in the clinical trials), subgroup analysis will be conducted relevant to these categories.

## 4 Discussion

As the COVID-19 is gradually brought under control, asymptomatic infections of COVID-19 are also becoming a new concern. They may also become the contagious source of novel coronavirus, and have risk of transmission. Asymptomatic infections also brought great threat to public and society. Acupuncture is a kind of important traditional Chinese medicine treatment with simple operation and low cost. Some Chinese hospitals are using acupuncture therapy to treat asymptomatic infections of COVID-19. If the evidence could prove acupuncture is useful for asymptomatic infections of COVID-19, it might save many costs and be beneficial to worldwide people. However, no systematic reviews on this topic have been published. In order to give compelling evidence and better guide in clinic practice, all actions of this review will be performed according to Cochrane Handbook 5.2.0.

## Author contributions

**Conceptualization:** Shaolei Huang, Dianhui Yang, Suyao Wang.

**Data curation:** Mengmeng Wang, Wenjie Yu, Shaolei Huang, Suyao Wang.

**Investigation:** Guoqiang Li, Guoliang Shao.

**Methodology:** Shaolei Huang, Jian Zhang.

**Supervision:** Shaolei Huang, Suyao Wang.

**Validation:** Dianhui Yang, Jian Zhang.

**Visualization:** Shaolei Huang.

**Writing – original draft:** Shaolei Huang, Suyao Wang.

**Writing – review & editing:** Dianhui Yang, Jian Zhang.
